# Analysis of Agricultural Biomass Energy Use and Greenhouse Gas Reduction Evidence from China

**DOI:** 10.1155/2022/6126944

**Published:** 2022-07-11

**Authors:** Deming Li

**Affiliations:** School of Economics and Management, Beijing Information Science and Technology University, Beijing, China

## Abstract

China is a large agricultural country, where agricultural activities and rural life cause a large amount of greenhouse gas (GHG) emissions. In the process of crop growth, production, and processing, a large number of crop straws and agricultural wasted products are produced, which become one of the important sources of biomass resources. However, few detailed studies focused on the potential of China's agricultural biomass energy conversion and carbon emission reduction, and fewer studies proposed GHG emission reduction strategies from the perspective of making full use of China's agricultural waste resources. In this study, the quantity calculation index of agricultural biomass energy was given, and the GHG emission reduction potential calculation index of agricultural biomass energy was constructed, with which the amount of GHG emissions caused by agricultural waste use in China was measured and the potential of GHG emission reduction caused by agricultural waste use would be easily speculated. Based on the statistical data of China, the quantity and GHG emission reduction potential of agricultural biomass resources in China in the recent 10 years (2009∼2018) were clarified. According to the research, the amount of agricultural waste equivalent to standard coal in China from 2009 to 2018 reached 280,0711 million tons. If all these resources were used to replace coal, a total of 4,474,483 million tons of carbon dioxide emissions could be saved. Assuming that these wastes are anaerobic, carbonized, or fully burned as fuel, CH_4_ emissions could be reduced by up to 12.024 million tons and N_2_O emissions by up to 185,000 tons. It can be seen that the effective utilization of agricultural biomass resources can replace coal, reduce backwardness such as land burning, and then reduce CO_2_, CH_4_, N_2_O, and other greenhouse gas emissions, and promote the realization of carbon peak and carbon neutrality.

## 1. Introduction

Since industrialization, the impact of global warming on natural and human systems has become increasingly significant. Scientists generally agree that more than 90% of the causes of global warming come from GHG emissions produced by human activities. Globally recognized GHG include carbon dioxide (CO_2_), methane (CH_4_), nitrous oxide (N_2_O), hydrofluorocarbons (HFCs), perfluorocarbons (PFCs), and sulfur hexafluoride (SF_6_). Among them, CO_2_ has been widely recognized as a major contributor to global warming. However, methane is the second largest GHG next to CO_2_, contributing 18% to global warming. From the perspective of global warming potential (GWP), methane's potential is 25 times that of CO_2_. The Paris Agreement proposed to limit global warming to 2°C and strived to limit global warming to 1.5°C in order to avoid the more severe effects of climate change. To further refine the strategic objectives of the Paris Agreement, the 26^th^ UN Climate Change Conference of the Parties (COP26), held in October 2021, was not only to sign a consensus but also to increase the intensity of more actions. In COP26, experts point out that international climate action can be considered as slowly entering deep waters, slowly involving all aspects of each country's political and economic energy system, and becoming a topic with real impact on each country. Therefore, controlling emissions of key greenhouse gases such as carbon dioxide and methane is a necessary condition to keep global warming below 1.5°C [1]. Building and operating more sustainable energy systems is an important measure to mitigate climate change [2].

According to global renewable energy data released by IRENA [3], renewables accounted for 26.2 percent of the world's electricity generation at the end of 2018 and about 18.1 percent of global primary energy consumption. As one kind of all renewable energies, biomass is the earliest energy used in human history, and its effective use will play a strong supporting role in the realization of China's carbon emission reduction and carbon peak goal [4]. The so-called biomass energy means that solar energy stores CO_2_ through photosynthesis and converts it into chemical energy in living matter, that is, energy with biomass as the carrier. It is directly or indirectly derived from the photosynthesis of green plants and can be converted into conventional solid, liquid, and gaseous fuels. It is inexhaustible and is the only renewable carbon source. Biomass energy can be widely used in industry, agriculture, transportation, civil life, and other fields through power generation, such as heat supply, gas supply, and other ways. The wide use of biomass energy will lead to the great potential of GHG emission reductions [5, 6]. At the same time, combined with carbon capture and storage (CCS) technology [7], biomass can absorb more carbon dioxide, thus creating carbon negative emissions [8]. Jiang et al. [9] believe that under the 1.5°C scenario, BECCS will increase rapidly after 2030, and over 820 million tons of CO_2_ will need to be removed annually by 2050. It has been calculated that biomass stores twice as much energy as the world currently consumes. The Biomass Industry Branch of the China Industrial Development Promotion Association recently released the “3060 Zero-carbon biomass Energy Development Potential Blue Book” (hereinafter referred to as the Blue Book). The Blue Book predicts that by 2030, biomass energy use will save more than 900 million tons of carbon for the whole society, and by 2060, it will achieve more than 2 billion tons of carbon reduction. Therefore, biomass energy not only has the attribute of zero carbon energy but also has the function of CCS. Biomass CCS technology is expected to stabilize global warming at a low level in the future. The IPCC points out that, historically, economic development has been closely associated with the increases in energy use and GHG emissions, while renewable energy can help break away from this correlation and thus contribute to sustainable development. It was found that increasing the proportion of biomass energy in all energy sources will promote economic development and reduce carbon dioxide emissions [10]. And the relationship between GHG emissions and energy consumption has been widely examined [11]. Biomass energy has significant potential to reduce GHG emissions if resources are sustainably developed and efficient technologies are used. Biomass energy sources are extensive, including agricultural waste resources, forest resources, livestock and poultry waste resources, organic wastewater resources, and urban household waste resources. Many scholars have calculated and predicted the amount of biomass energy in the world [12, 13], and IPCC [14] estimated that the maximum theoretical potential of global biomass energy was about 1500EJ/*a*, and the maximum potential of global biomass energy technology could reach 500EJ/*a* by 2050. Considering socioeconomic development, climate change, and limitations of land freshwater and biodiversity, the potential extension and utilization level of biomass that can be used for energy utilization in 2050 is between 100 and 300 EJ/*a*.

Agriculture is now one of the main sources of global GHG emissions, accounting for about a fifth of global emissions. China is a big country in agricultural production. A large number of crop straws and agricultural products processing wastes are generated in the life cycle of crop growth, production, and processing, which makes China have a stable agricultural biomass resource base. It is of great significance to make good use of agricultural biomass resources to achieve dual goals of carbon emission reduction and carbon peak and to provide stable and high-quality rural energy. Research shows that farmers can use the waste from crop cultivation and production as energy to meet the needs of mechanical equipment such as tractors [15, 16]. Agricultural waste is also proposed to be used from the perspective of a circular economy [17]. Energy generation potential from different kinds of main crops and agricultural byproducts, like rice straw, sugar can straw, and coffee husks, has been well calculated by researchers [18], which is diversified across all the countries. Some experts also have achieved long-term forecasts of biomass energy potential across China from 2020 to 2100 [19]. China's rural energy consumption is mainly based on biomass energy such as straws and fuelwood, which are easy to obtain locally. According to the Food and Agriculture Organization of the United Nations (FAO), agricultural land releases more than 30% of the world's total anthropogenic greenhouse gas emissions, equivalent to generating 15 billion tons of carbon dioxide per year. It is worth noting that GHG emissions from agricultural sources still account for 24% of China's total GHG emissions, of which methane and nitrous oxide emissions from agricultural activities in China account for 40% and 60%. Therefore, adjusting the agricultural structure and developing and promoting low-carbon emission reduction production technologies are not only the practical needs for alleviating global climate change but also the strategic choice for China to maintain sustainable agricultural development and accelerate the realization of “carbon peak” and “carbon neutrality.” The traditional utilization of biomass energy accounts for about 1/3 of the total energy consumption in China's rural areas. In the vast rural areas of China, a considerable part of the crop wastes is used as fuel, mainly including wheat straw, rice straw, corn straw, and cotton straw. Therefore, the burning of this part of crop straw becomes one of the main emission sources of CO_2_. In addition, returning crop straw to the field is also one of the emission sources of methane and nitrous oxide.

In summary, the existing research has laid a good theoretical and methodological foundation for this paper. However, under the severe situation of carbon dioxide emission reduction, China is an important committed country of the Paris Agreement, whose emission reduction potential and emission reduction efforts will make an important contribution to the achievement of global carbon emission reduction targets. China has a vast rural area and abundant agricultural waste resources. However, there are few detailed studies that have focused on the potential of China's agricultural biomass energy conversion and carbon emission reduction, and fewer studies have proposed GHG emission reduction strategies from the perspective of making full use of China's agricultural waste resources. Therefore, measuring and mastering the amount of GHG emissions caused by agricultural waste use in China becomes the basis for making full use of agricultural biomass energy and controlling GHG emissions.

## 2. Data Collection and Methods

### 2.1. Mechanism Analysis of GHG Emission Reduction of Agricultural Waste Biomass Resources

Crop straw is mainly carbohydrate, in addition to containing a small amount of nitrogen, phosphorus, and other nutrients. Theoretically speaking, the combustion process is a full oxidation process, and its products should be carbon dioxide and water. However, in the actual combustion process, the oxygenation process is not sufficient. In incomplete combustion, the combustion products of agricultural straw contain a certain amount of reducing products, such as methane, nitrous oxide, etc. In particular, in rural China, land reclamation is generally accompanied by incomplete combustion processes, which increase methane and nitrous oxide emissions. In summary, the mechanism of GHG emission reduction by energy utilization of agricultural waste biomass resources in China is mainly reflected in the following paths:

1. Carbon sequestration. Plant biomass resources absorb CO_2_ from the atmosphere during their growth and become carbon sinks.
2. Anaerobic emission reduction. Anaerobic treatment of straw, weeds, livestock and poultry waste, and organic waste water can reduce the direct emission of CH_4_ into the atmosphere.
3. Anaerobic treatment to achieve emission reduction. Biomass energy substitutes fossil fuel combustion, forms carbon source, and releases relatively fewer GHGs.
4. Clean energy. As a clean fuel, agricultural biomass energy can be used for power generation, heating, or household cooking energy, which can replace coal utilization and reduce CO_2_ emissions from coal combustion to meet the same energy demand.

Since path (1) and path (3) are mutually inverse processes, the two paths will be ignored in the following calculation of this research. The subsequent calculation of GHG emission reduction potential only includes paths (2) and (4).

### 2.2. Resources and Reserves of Agricultural Wastes in China

#### 2.2.1. Evaluation Index of Agricultural Waste Resource Reserves

Based on the comprehensive research, the present research selected theoretical resources quantity (TRQ) and collectable resources quantity (CRQ) as the measurement indexes of Agricultural waste resources in China.

*(1). Theoretic Resources Quantity*. TRQ refers to the annual total output of agricultural waste calculated according to the agricultural crop yield and straw-valley ratio in a certain region, that is, the annual total output of crop straws calculated according to the crop yield and straw-valley ratio, indicating the theoretical amount of straw resources that could be produced in the specific region every year.

(1) TRQ=∑i=1nPλii,

where TRQ is the total theoretical amount of agricultural waste resources produced in the region; *Pi* is the seed yield of a particular crop *i*; *λi* is the output coefficient of straw and other agricultural waste resources relative to seed yield.

*(2) Collectable Resources Quantity*. CRQ refers to the amount of agricultural waste resources collected in a certain region through all the existing collection methods. It is generally measured by TRQ and collectable coefficient.

(2) $$\begin{array}{c} \text{CRQ}=\sum_{i=1}^{n}TRQ_{i}\eta_{i}, \end{array}$$

where CRQ is collectable resource quantity in a specific region, and *η*_*i*_ represents the collectable coefficient relative to *TRQ*_*i*_.

#### 2.2.2. Related Coefficients

*(1). Output coefficient*. In this paper, resource output coefficient mainly refers to crop straw output coefficient, that is, the ratio of crop straw yield to grain yield per unit area, as shown in Table 1.

*(2). Collectable coefficient*. Crop straw is a dispersed resource with poor collection rate, which will change with industrial developments. Resource collectable coefficient refers to the proportion of certain crop straw in the total theoretical output of resources in a certain region, which is an important index in the estimation of resource quantity. The specific estimation can be based on crop stubble height and total plant height, but there are differences in straw collectable coefficient due to different stubble height of different harvesting methods. Different harvesting methods should be taken into account when evaluating the collection rate of certain crop straw.

(3) $$\begin{array}{c} \eta_{i,s}=\sum \alpha_{j}\beta_{j}, \end{array}$$

where *η*_*i*_ is the collectable coefficient considering the harvesting method and the ratio of different methods used for crop *j*. *α*_*j*_ is the coefficient of the harvest method, and *β*_*j*_ represents the ratio of *α*_*j*_ that can be used. At present, mechanical harvesting is only widely applied in wheat, rice, corn, and cotton in China, while the mechanical harvesting rate of soybean, peanut, sesame, and other crops is low, less than 10% or lower, which can be ignored. Therefore, in this study, only four crops of wheat, rice, corn, and cotton wasted stem were calculated according to different harvesting methods, as shown in Table 2.

*(3). Standard coal coefficient*. As the composition of agricultural waste is diverse, even the calorific value of the same category of waste is very different. For the convenience of the following calculation, CRQ for different kinds of agricultural wastes can be converted into the quantity of standard coal, as shown in Table 3.

### 2.3. Calculation Methods for GHG Emission Reduction Potential

#### 2.3.1. Calculation Method for CO_2_ Emission by Using Agricultural Waste Biomass Energy

On the basis of converting agricultural waste biomass resources into standard coal quantity, the CO_2_ emission reduction potential of agricultural waste biomass resources can be calculated through the CO_2_ calculation formula of coal burning. The calculation formula is as follows:

(4) $$\begin{array}{c} C_{\text{coal}}=C\times \left(C_{p}-C_{s}\right)\times C_{o}\times \frac{44}{12}, \end{array}$$

where *C*_coal_ is the amount of CO_2_ emission from coal burning in tons, *C* is the amount of coal consumption in tons, *C*_*P*_ represents the amount of carbon in the burning fuel expressed in percentage, *C*_*S*_ is the amount of carbon sequestration of fuel, in percentage, *C*_*O*_ is Oxidation rate of carbon, expressed in percentage, and 44/12 is the ratio of the molecular mass of CO_2_ to the atomic mass of carbon。Product carbon sequestration refers to the carbon not emitted or not immediately emitted when fuel is used for nonenergy purposes, which can be ignored in energy consumption. Based on the calculation of the amount of agricultural waste converted into standard coal, the amount of carbon dioxide emitted by the direct combustion of agricultural waste as fuel can be obtained.

#### 2.3.2. Calculations of CH_4_ and N_2_O Emissions from Agricultural Biomass Energy Consumption

According to the calculation method of IPCC [20], firstly, the total amount of carbon burned in agricultural biomass resources (*C*_*abr*_) is calculated. Secondly, the total amount of methane and nitrous oxide is calculated based on the total amount of carbon combustion. The specific calculation formula is as follows:

(5) $$\begin{array}{c} C_{\text{coal}}=\sum_{i}^{n}CRQ_{i}\times B_{i}\times C_{i}, \end{array}$$

(6) $$\begin{array}{c} {\text{CH}}_{4}-C_{\text{emission}}\left(\text{low}\right)=C_{\text{coal}}\times 0.9\times 0.007, \end{array}$$

(7) $$\begin{array}{c} {\text{CH}}_{4}-C_{\text{emission}}\left(\text{high}\right)=C_{\text{coal}}\times 0.9\times 0.013, \end{array}$$

(8) $$\begin{array}{c} {\text{N}}_{2}\text{O}-N_{\text{emission}}\left(\text{low}\right)=C_{\text{coal}}\times 0.1\times 0.005, \end{array}$$

(9) $$\begin{array}{c} {\text{N}}_{2}\text{O}-N_{\text{emission}}\left(\text{high}\right)=C_{\text{coal}}\times 0.2\times 0.009, \end{array}$$

where *B* is the percentage of straw burning, DM is the percentage of dry matter of agricultural biomass resource *i*, and C represents the percentage of carbon of agricultural biomass resource *i*.

#### 2.3.3. Data

This study mainly relied on the statistical data in China Statistical Yearbook 2019, with which the number of agricultural waste resources in China from 2009 to 2018 was estimated according to the calculation methods mentioned above. In this study, the focus is on the analysis and estimation of the GHG emission reduction potential of major crops and their waste, specifically involving wheat straw, rice straw, corn straw, and cotton straw [21]. Crop yield data come from China Statistical Yearbook and China Agricultural Statistics.

## 3. Results

### 3.1. Total Agricultural Biomass Resources in China

Based on the above data and the calculation methods, the amount of China's four key crop resources in 2018 was calculated. The specific data are shown in Table 4 and Figure 1. Among them, the theoretical resource quantity of agricultural waste biomass resources is 694.109 million tons, and the actual collectable resource quantity that can be collected is 610.816 million tons.

As shown in Table 5 and Figure 2, the total amount of recyclable agricultural wastes in China has an obvious trend of gradual increase, especially cotton and rice wastes.

In 2018, the TRQ of agricultural waste in China was about 6.94 × 10^8^ tons of standard coal, and the CRQ was about 6.11 × 10^8^ tons of standard coal. As shown in Table 6, the quantity trend of agricultural waste converted into standard coal from 2009 to 2018 reached 280,0711 million tons. For more specific data, please see Tables 6 and 7.

### 3.2. GHG Emission Reduction Benefits of Agricultural Biomass Resources in China

According to the analysis of the GHG emission reduction mechanism of agricultural waste biomass resources in Section 2.1, this paper will study the GHG emission reduction effectiveness of Biomass resources in China from the perspective of CO_2_ emission reduction benefits and CH_4_ and N_2_O emission reduction benefits.

#### 3.2.1. The Potential CO_2_ Reduction Benefits

As a clean fuel, biomass energy can be used for power generation, heating, or cooking for residents. It can replace coal utilization and reduce CO_2_ emissions from coal combustion to meet the same energy demand. It is assumed in this study that the production and processing wastes of rice, wheat, corn, and cotton in China are all used to replace coal burning. Based on the principle of converting different energy sources into the same standard coal, the actual amount of coal that can be replaced by agricultural waste biomass resources in China from 2009 to 2018 can be calculated, as shown in Table 6. If all agricultural biomass resources in China were used to replace coal from 2009 to 2018, a total of 44.75 × 10^8^ tons of CO_2_ emissions could be reduced, as shown in Table 8.

#### 3.2.2. The Potential CH_4_ and N_2_O Reduction Benefits

The anaerobic treatment of agricultural wastes such as straw reduces the direct emission of CH_4_ into the atmosphere. At the same time, the agricultural waste is carbonized or burned as fuel to avoid the emission of methane and nitrous oxide in the process of burning waste and returning waste to the land. According to formula (5)–(9), it is assumed that the four major agricultural wastes of rice, wheat, corn, and cotton in China are anaerobic, carbonized, or fully burned as fuel. From 2009 to 2018, the methane emission can be reduced by 12.024 million tons and nitrous oxide emissions by 185,000 tons at most. The specific results are shown in Table 9.

## 4. Discussion

Based on the statistical data of China, the quantity and GHG emission reduction potential of agricultural biomass resources in China in the recent 10 years (2009∼2018) were analyzed above. In recent 10 years, agricultural waste biomass resources in China presented a slow growth and a steady development trend. With the advancement of agricultural mechanization, the degree of mechanization of crop harvesting has gradually improved, and the number of stubble left by mechanized harvesting has also gradually increased, which makes the agricultural biomass resources that can be used (CRQ) reduce. According to the analysis, the amount of agricultural CRQ equivalent to standard coal in China from 2009 to 2018 reached 280,0711 million tons. It can be seen that the amount of corn, rice, wheat planting, and production wastes converted into standard coal is relatively high. However, in terms of the total amount, the change rate of agricultural waste converted into standard coal is not obvious. Compared with 1978, their annual growth rates were 2.18% and 2.19%, respectively.

If all these resources were used to replace coal, a total of 4,474,483 million tons of carbon dioxide emissions could be saved. Assuming that these wastes are anaerobic, carbonized, or fully burned as fuel, CH_4_ emissions could be reduced by up to 12.024 million tons and N_2_O emissions by up to 185,000 tons. It can be seen that the effective utilization of agricultural biomass resources can replace coal, reduce backwardness such as land burning, and then reduce CO_2_, CH_4_, N_2_O, and other greenhouse gas emissions, and promote the realization of carbon peak and carbon neutrality.

## 5. Conclusions

The present paper investigated the amount of agricultural biomass energy and the potential benefits of CO_2_, CH_4,_ and N_2_O emission reductions in China from 2009 to 2018. The research shows that through rational and effective utilization of agricultural waste biomass resources, it can realize the effective replacement of coal resources, realize the improvement of backward production and life style, and then realize the reduction of GHG, which has significant social and environmental benefits. According to the research results, from 2009 to 2018, the amount of agricultural waste equivalent to standard coal in China reached 280,0711 million tons. If all these resources were used to replace coal, a total of 4,474,483 million tons of CO_2_ emissions could be saved. Assuming that these wastes are anaerobic, carbonized, or fully burned as fuel, CH_4_ emissions could be reduced by up to 12.024 million tons and N_2_O emissions by 185,000 tons. Therefore, strengthening the effective development and utilization of agricultural waste biomass resources in China will play an effective role in promoting the realization of carbon neutrality and carbon peak.

In order to better realize the development and utilization of agricultural biomass energy in rural China, this study puts forward the following policy recommendations.

First of all, improve the policy and regulation system for the development and utilization of agricultural waste biomass energy and increase capital investment.

Second, further popularize rural biogas, biomass power generation, and other renewable energy and reduce the traditional treatment of straw. In areas with abundant solar energy resources and suitable climate conditions, more solar water heaters and solar houses should be developed to effectively solve the problem of heating and electricity consumption in rural areas.

Third, promote the construction of agricultural biomass resource collection, transportation, and recycling systems. The construction of the system needs to fully consider the differences between various provinces in China, such as the differences in crop resources, energy systems, and the present status of infrastructure.

Finally, based on the carbon sequestration characteristics of agricultural waste biomass resources, BECCS negative carbon emission technology is suggested to be developed and deployed in advance.

## Figures and Tables

**Figure 1:** Total amount of agricultural biomass resources in China, 2018.

**Figure 2:** Total amount of collectable agricultural biomass resources in China, 2018.

**Table 1:** Output coefficients of crop straw and agricultural product processing in China.

Crop	*λ*
Wheat stem	1.17
Corn stem	1.04
Cotton stem	3.00
Rice stem	1.00

**Table 2:** Stubble height of four main crops harvested in different ways.

Crop	Harvesting methods	Plant height (cm)	Stubble height	*αj*	*βj*
Wheat	Artificial harvesting	85	6	0.93	0.83
	Mechanized harvesting		25	0.71	0.73

Rice	Artificial harvesting	100	7	0.93	0.83
	Mechanized harvesting		16	0.84	0.74

Corn	Artificial harvesting	250	6	0.98	0.85
	Mechanized harvesting		15	0.94	0.90

Cotton	Artificial harvesting	100	6	0.93	0.82
	Mechanized harvesting		10	0.95	0.86

Source: Ministry of agriculture, PRC.

**Table 3:** Standard coal coefficient of agricultural waste (kg Standard coal/kg).

Crop	Standard coal coefficient
Rice stem	0.429
Wheat stem	0.500
Corn stem	0.529
Cotton stem	0.543

**Table 4:** Total amount of agricultural biomass resources in China, 2018.

Crop type	Area (10^3^ hectares)	Total production (10^4^ t)	TRQ (10^4^ t)	CRQ (10^4^ t)
Rice	30189	21212.9	25455.5	22400.8
Wheat	13144	13144	15378.5	13533.1
Corn	25717.4	25717.4	26746.1	23536.6
Cotton	3354	610.3	1830.8	1611.1

**Table 5:** Total amount of collectable agricultural biomass resources in China, 2009∼2018.

Year	2009	2010	2011	2012	2013
Rice	20718.4	20827	21424.4	21809.8	21783.8

Wheat	11926.3	11957.9	12213.7	12616.7	12737.2

Corn	15856.6	17457.6	19339.6	21009.2	22738.4

Cotton	1646.3	1523.4	1721	1744.5	1658.3

Year	2014	2015	2016	2017	2018

Rice	22134.7	22402.2	22291.6	22458.6	22400.8

Wheat	13211.9	13656.5	13721.5	13831	13533.1

Corn	22858.4	24252.1	24125.9	23710.2	23536.6

Cotton	1663.1	1559.6	1410.5	1492.4	1611.1

**Table 6:** The sown area and yield of major crops in China, 2009∼2018.

Year	Rice		Wheat		Corn		Legume crops		Tuber crops		Cotton		Rapeseed		Sugarcane	
	Plant area (10^3^ hectares)	Output (10^4^ tons)	Plant area (10^3^ hectares)	Output (10^4^ tons)	Plant area (10^3^ hectares)	Output (10^4^ tons)	Plant area (10^3^ hectares)	Output (10^4^ tons)	Plant area (10^3^ hectares)	Output (10^4^ tons)	Plant area (10^3^ hectares)	Output (10^4^ tons)	Plant area (10^3^ hectares)	Output (10^4^ tons)	Plant area (10^3^ hectares)	Output (10^4^ tons)
2009	29793	19619.7	24442	11583.4	32948	17325.9	11785	1904.6	8088	2792.9	4485	623.6	7170	1353.6	1643	11200.4
2010	30097	19722.6	24459	11614.1	34977	19075.2	11053	1871.8	8021	2842.7	4366	577.0	7316	1278.8	1624	10598.2
2011	30338	20288.3	24523	11862.5	36767	21131.6	10367	1863.3	7998	2924.3	4524	651.9	7192	1313.7	1644	10867.4
2012	30476	20653.2	24576	12254.0	39109	22955.9	9405	1680.6	7821	2883.0	4360	660.8	7187	1340.1	1696	11574.6
2013	30710	20628.6	24470	12371.0	41299	24845.3	8893	1542.4	7727	2855.4	4162	628.2	7193	1352.3	1704	11926.4
2014	30765	20960.9	24472	12832.1	42997	24976.4	8824	1564.5	7544	2798.8	4176	629.9	7158	1391.4	1638	11578.8
2015	30784	21214.2	24596	13263.9	44968	26499.2	8433	1512.5	7305	2729.3	3775	590.7	7028	1385.9	1476	10706.4
2016	30746	21109.4	24694	13327.0	44178	26361.3	9287	1650.7	7241	2726.3	3198	534.3	6623	1312.8	1402	10321.5
2017	30747	21267.6	24508	13433.4	42399	25907.1	10051	1841.6	7173	2798.6	3195	565.3	6653	1327.4	1371	10440.4
2018	30189	21212.9	24266	13144.0	42130	25717.4	10186	1920.3	7180	2865.4	3354	610.3	6551	1328.1	1406	10809.7

Source: China Statistical Yearbook, 2019.

**Table 7:** Total amount of collectable agricultural resources and alternative coal in China, 2009∼2018.

Year	Rice			Wheat			Corn			Cotton			Total amount of the four kinds of biomass resources		
	TRQ (10^4^* *t)	CRQ (10^4^* *t)	Alternative coal (10^4^* *t)	TRQ (10^4^* *t)	CRQ (10^4^* *t)	Alternative coal (10^4^* *t)	TRQ (10^4^* *t)	CRQ (10^4^* *t)	Alternative coal (10^4^* *t)	TRQ (10^4^* *t)	CRQ (10^4^* *t)	Alternative coal (10^4^* *t)	TRQ (10^4^* *t)	CRQ (10^4^* *t)	Alternative coal (10^4^* *t)
2009	23543.6	20718.4	8888.2	13552.6	11926.3	5963.1	18018.9	15856.6	8388.2	1870.8	1646.3	893.9	56985.8	50147.5	24133.4
2010	23667.1	20827	8934.8	13588.5	11957.9	5978.9	19838.2	17457.6	9235.1	1731.1	1523.4	827.2	58824.9	51765.9	24976
2011	24345.9	21424.4	9191.1	13879.2	12213.7	6106.8	21976.9	19339.6	10230.7	1955.7	1721	934.5	62157.6	54698.7	26463.1
2012	24783.9	21809.8	9356.4	14337.2	12616.7	6308.3	23874.1	21009.2	11113.9	1982.4	1744.5	947.3	64977.6	57180.3	27725.9
2013	24754.3	21783.8	9345.2	14474.1	12737.2	6368.6	25839.1	22738.4	12028.6	1884.5	1658.3	900.5	66952	58917.7	28643
2014	25153.1	22134.7	9495.8	15013.5	13211.9	6606	25975.5	22858.4	12092.1	1889.8	1663.1	903	68032	59868.1	29096.9
2015	25457	22402.2	9610.5	15518.8	13656.5	6828.3	27559.2	24252.1	12829.4	1772.2	1559.6	846.8	70307.2	61870.4	30115
2016	25331.3	22291.6	9563.1	15592.6	13721.5	6860.8	27415.8	24125.9	12762.6	1602.9	1410.5	765.9	69942.6	61549.5	29952.3
2017	25521.1	22458.6	9634.7	15717.1	13831	6915.5	26943.4	23710.2	12542.7	1695.9	1492.4	810.4	69877.4	61492.1	29903.3
2018	25455.5	22400.8	9610	15378.5	13533.1	6766.6	26746.1	23536.6	12450.8	1830.8	1611.1	874.8	69410.9	61081.6	29702.2

**Table 8:** Benefits of CO_2_ reduction by using agricultural biomass energy in China, 2009∼2018.

Year	Alternative coal (10^4^ t)	CO_2_ emission reductions (10^4^ t)
2009	26142.4	38881.58455
2010	26986	40136.2706
2011	28474.1	42349.52134
2012	29737.9	44229.17074
2013	30655.9	45594.5119
2014	31110.9	46271.23327
2015	32130	47786.94043
2016	31968.4	47546.5928
2017	31920.3	47475.05368
2018	31720.2	47177.445
Total	300846.1	447448.3243

**Table 9:** Benefits of CH_4_-C emission and N_2_O emission reduction by using agricultural biomass energy in China, 2009∼2018.

Item		Rice	Wheat	Corn	Cotton
Percentage of straw burning (%)		0.60	0.60	0.60	0.60
Percentage of dry matter (%)		0.83	0.83	0.40	0.50
Percentage of carbon (%)		0.41	0.49	0.47	0.45

2009	Physical resources quantity (10^4^ t)	20718.40	11926.30	15856.60	1646.30
	Total amount of carbon burned (10^4^ t)	4275.68	2882.34	1792.05	222.25
	CH_4_-C emission (Low) (10^4^ t)	26.94	18.16	11.29	1.40
	CH_4_-C emission (High) (10^4^ t)	50.03	33.72	20.97	2.60
	N_2_O emission (Low) (10^4^ t)	0.21	0.14	0.09	0.01
	N_2_O emission (High) (10^4^ t)	0.77	0.52	0.32	0.04

2010	Physical resources quantity (10^4^ t)	20827.00	11957.90	17457.60	1523.40
	Total amount of carbon burned (10^4^ t)	4298.09	2889.98	1972.99	205.66
	CH_4_-C emission (Low) (10^4^ t)	27.08	18.21	12.43	1.30
	CH_4_-C emission (High) (10^4^ t)	50.29	33.81	23.08	2.41
	N_2_O emission (Low) (10^4^ t)	0.21	0.14	0.10	0.01
	N_2_O emission (High) (10^4^ t)	0.77	0.52	0.36	0.04

2011	Physical resources quantity (10^4^ t)	21424.40	12213.70	19339.60	1721.00
	Total amount of carbon burned (10^4^ t)	4421.38	2951.80	2185.68	232.34
	CH_4_-C emission (Low) (10^4^ t)	27.85	18.60	13.77	1.46
	CH_4_-C emission (High) (10^4^ t)	51.73	34.54	25.57	2.72
	N_2_O emission (Low) (10^4^ t)	0.22	0.15	0.11	0.01
	N_2_O emission (High) (10^4^ t)	0.80	0.53	0.39	0.04

2012	Physical resources quantity (10^4^ t)	21809.80	12616.70	21009.20	1744.50
	Total amount of carbon burned (10^4^ t)	4500.91	3049.20	2374.38	235.51
	CH_4_-C emission (Low) (10^4^ t)	28.36	19.21	14.96	1.48
	CH_4_-C emission (High) (10^4^ t)	52.66	35.68	27.78	2.76
	N_2_O emission (Low) (10^4^ t)	0.23	0.15	0.12	0.01
	N_2_O emission (High) (10^4^ t)	0.81	0.55	0.43	0.04

2013	Physical resources quantity (10^4^ t)	21783.80	12737.20	22738.40	1658.30
	Total amount of carbon burned (10^4^ t)	4495.55	3078.32	2569.80	223.87
	CH_4_-C emission (Low) (10^4^ t)	28.32	19.39	16.19	1.41
	CH_4_-C emission (High) (10^4^ t)	52.60	36.02	30.07	2.62
	N_2_O emission (Low) (10^4^ t)	0.22	0.15	0.13	0.01
	N_2_O emission (High) (10^4^ t)	0.81	0.55	0.46	0.04

2014	Physical resources quantity (10^4^ t)	22134.70	13211.90	22858.40	1663.10
	Total amount of carbon burned (10^4^ t)	4567.96	3193.04	2583.36	224.52
	CH_4_-C emission (Low) (10^4^ t)	28.78	20.12	16.28	1.41
	CH_4_-C emission (High) (10^4^ t)	53.45	37.36	30.23	2.63
	N_2_O emission (Low) (10^4^ t)	0.23	0.16	0.13	0.01
	N_2_O emission (High) (10^4^ t)	0.82	0.57	0.47	0.04

2015	Physical resources quantity (10^4^ t)	22402.20	13656.50	24252.10	1559.60
	Total amount of carbon burned (10^4^ t)	4623.17	3300.49	2740.88	210.55
	CH_4_-C emission (Low) (10^4^ t)	29.13	20.79	17.27	1.33
	CH_4_-C emission (High) (10^4^ t)	54.09	38.62	32.07	2.46
	N_2_O emission (Low) (10^4^ t)	0.23	0.17	0.14	0.01
	N_2_O emission (High) (10^4^ t)	0.83	0.59	0.49	0.04

2016	Physical resources quantity (10^4^ t)	22291.60	13721.50	24125.90	1410.50
	Total amount of carbon burned (10^4^ t)	4600.34	3316.20	2726.61	190.42
	CH_4_-C emission (Low) (10^4^ t)	28.98	20.89	17.18	1.20
	CH_4_-C emission (High) (10^4^ t)	53.82	38.80	31.90	2.23
	N_2_O emission (Low) (10^4^ t)	0.23	0.17	0.14	0.01
	N_2_O emission (High) (10^4^ t)	0.83	0.60	0.49	0.03

2017	Physical resources quantity (10^4^ t)	22458.60	13831.00	23710.20	1492.40
	Total amount of carbon burned (10^4^ t)	4634.81	3342.67	2679.63	201.47
	CH_4_-C emission (Low) (10^4^ t)	29.20	21.06	16.88	1.27
	CH_4_-C emission (High) (10^4^ t)	54.23	39.11	31.35	2.36
	N_2_O emission (Low) (10^4^ t)	0.23	0.17	0.13	0.01
	N_2_O emission (High) (10^4^ t)	0.83	0.60	0.48	0.04

2018	Physical resources quantity (10^4^ t)	22400.80	13533.10	23536.60	1611.10
	Total amount of carbon burned (10^4^ t)	4622.88	3270.67	2660.01	217.50
	CH_4_-C emission (Low) (10^4^ t)	29.12	20.61	16.76	1.37
	CH_4_-C emission (High) (10^4^ t)	54.09	38.27	31.12	2.54
	N_2_O emission (Low) (10^4^ t)	0.23	0.16	0.13	0.01
	N_2_O emission (High) (10^4^ t)	0.83	0.59	0.48	0.04

## Data Availability

All data used in the study can be accessed by request.
